# Intelligent Classification Method of Archive Data Based on Multigranular Semantics

**DOI:** 10.1155/2022/7559523

**Published:** 2022-05-14

**Authors:** Xiaobo Jiang

**Affiliations:** Jilin University of Architecture and Technology, Changchun, Jilin 130114, China

## Abstract

With the rapid development of information technology, the amount of data in various digital archives has exploded. How to reasonably mine and analyze archive data and improve the effect of intelligent management of newly included archives has become an urgent problem to be solved. The existing archival data classification method is manual classification oriented to management needs. This manual classification method is inefficient and ignores the inherent content information of the archives. In addition, for the discovery and utilization of archive information, it is necessary to further explore and analyze the correlation between the contents of the archive data. Facing the needs of intelligent archive management, from the perspective of the text content of archive data, further analysis of manually classified archives is carried out. Therefore, this paper proposes an intelligent classification method for archive data based on multigranular semantics. First, it constructs a semantic-label multigranular attention model; that is, the output of the stacked expanded convolutional coding module and the label graph attention module are jointly connected to the multigranular attention Mechanism network, the weighted label output by the multigranularity attention mechanism network is used as the input of the fully connected layer, and the output value of the fully connected layer used to map the predicted label is input into a Sigmoid layer to obtain the predicted probability of each label; then, the model for training: use the multilabel data set to train the constructed semantic-label multigranularity attention model, adjust the parameters until the semantic-label multigranularity attention model converges, and obtain the trained semantic-label multigranularity attention model. Taking the multilabel data set to be classified as input, the semantic-label multigranularity attention model after training outputs the classification result.

## 1. Introduction

With the development of China's digital archives construction, facing the massive digital archive data, simple statistical methods, or traditional data analysis cannot find the correlation between archive data. Manual classification, compilation, and research of archives also require a lot of manpower and material resources, which takes too long. Therefore, how to discover and use the hidden value of archive data to quickly and accurately classify massive digital archives is a major challenge facing the current archives management field [1–7].

The existing archival data management methods mostly rely on traditional database technology. The goal is to list and organize archival information and basic statistical analysis. The limitation of database management is that it requires artificial design and analysis content, and the people who formulate the analysis content are required to have a wealth of Experience support. With the rapid update of knowledge, traditional statistical analysis methods cannot meet the association of the content of the excavated archive data and cannot meet the requirements of higher-level intelligent management of archives. At present, natural language processing has become an important branch of artificial intelligence. Natural language processing can classify and cluster digital archives based on the content of digital archives and can well show the changes in the content of digital archives. Among the many association analysis methods, the method based on semantic features provides valuable reference for archive management. Therefore, mining the content of digital archives is the basis of intelligent archive management. In-depth analysis of the existing digital archive data can better understand the inherent association laws of different types of archives and predict the possible association relationships, so as to provide help for archive managers in archive association analysis and automatic classification [8–12].

Multilabel classification (MLC) is the task of assigning one or more labels to a given input sample. It has a wide range of application scenarios in the real world, such as document annotation, tag recommendation, information retrieval, and dialogue systems. Because the old tags usually have complex dependencies, this makes this task extremely challenging in the field of natural language processing.

Some early research work includes Binary Relevance (BR), Classifier Chains (CC), and Label Powerset (LP) that have achieved good results. As the deep learning based on artificial neural network has made great progress, people have begun to try to use the classic neural network architecture to deal with multilabel classification problems. For example, Zhang et al. used fully connected neural networks and paired ranking loss functions to handle multilabel classification tasks. The overall performance of these methods is to make People satisfied [13–18].

With sequence-to-sequence architecture and attention mechanism, great success has been achieved in neural machine translation tasks. Nam Yang, Lin, and others tried to use them for multilabel classification (MLC) tasks and achieved very advanced results. The sequence-to-sequence model based on attention mechanism uses RNN or long short-term memory network (LSTM) as the encoder to capture the context information in the input sequence, and the decoder also uses RNN or LSTM to generate the label sequence and predict the label. The application of the attention mechanism takes into account the contribution of different parts of the input sequence to the prediction of the label sequence.

The research topic of neural network has received more and more attention in recent years. It is proven to be able to effectively handle tasks with rich relational structures. Shi et al. proposed a multilabel graph convolutional network (ML-GCN) to achieve good results on the task of multilabel node classification. Lanchantin et al. proposed a label information transfer network (LaMP) based on the idea of message transfer in graph neural networks and achieved advanced results on multiple MLC tasks [19–23].

In some early studies, they did not fully consider the impact of the correlation between tags on the prediction of tags or did not fully consider the correlation between tags. For sequence models such as RNN or LSTM, the tag sequence can only be generated sequentially. This makes the sequence-to-sequence architecture limited in time efficiency. In addition, for specific MLC tasks, ideally, sequence factors cannot be considered between output tags. However, the label ranking of the above model is fixed during the training process (usually in descending order), which causes the model to often produce unstable predictions during testing, which reduces the performance and interpretability of the model. For the graph neural network model, only the relationship between the label and the sample is measured, and the influence of different content within the text on the prediction result is not considered, so it is difficult to apply it to other classic MLC tasks on a large scale [24–27].

Granularity is a tool for describing objects. It is a new concept and computing paradigm for information processing, and the theories, methods, techniques, and tools related to granularity are mainly used to establish a clear model for the intelligent processing of massive amounts of information. For the concept of granules, there is currently no precise definition for granules. From a certain perspective, granules can be regarded as blocks formed by certain relations, such as fuzzy relations, similar relations, and functional relations. People are limited to cognitive ability. When the information to be processed is very complex, the information is divided into information blocks based on logical structure and related relationships, and the information blocks obtained by the division are a granular concept. Within the scope of using the concept of granule, if a granule that cannot be subdivided is defined, it can be called a basic granule. If you use granules to describe files, the smallest unit of information can be called basic granules. As the smallest unit of describing the system, basic granules can be regarded as the most basic constituent elements.

When using the concept of granules, the research object can be divided into a system about granules according to the needs. In the system, there is a certain level of structure, that is, the level of granules, which can be called granularity. Different ways and degrees of granulation produce different levels of granulation systems. Taking a person's archive document as an example, it can be considered that the smallest information is fine-grained, columns are composed of information, tables are composed of columns, and the entire file is composed of tables; conversely, starting from the decomposing of the file, it can be divided into many tables. Granules have the properties of decomposition and assembly. The description of the problem can be carried out from different granularities. Fine granularity means that the granularity is more decomposed, which represents a more detailed description of the problem. On the contrary, coarse-grained means that the decomposition level is small, and it means that there is only a superficial description of the problem. According to the degree of decomposition of the granules, namely, the granularity, the granules can be divided into three levels of granularity: coarse granules, which are the largest parent granules; fine granules, which are basic granules and nondivisible granules; medium granules, which exist between coarse and coarse granules. The grains between the fine grains. Take a file as an example. The entire document is coarse-grained, and the content of a specific column is fine-grained. The part of the information between the coarse-grained and fine-grained can be considered as medium-grained.

In terms of operation and access to the knowledge element, the fine-grained one has advantages, but the operation of the entire document is not enough. The coarse-grained method has a good effect on the operation of the entire document, but for the mining of details, the in-depth knowledge element of processing is not ideal. Medium granularity is between coarse granularity and fine granularity. If a tree structure is used to describe the document, medium granularity is equivalent to information. In the retrieval system, fragments of this level can be returned. Compared with fine-grained, the medium-grained one saves space and time costs. Compared with coarse-grained, medium-grained method can operate on knowledge elements.

## 2. Intelligent Classification Method of Archive Data Based on Multigranular Semantics

As shown in Figure 1, this paper introduces a multilabel classification method based on semantic-label multigranularity attention. This article uses this method to apply to the server as an example. It is understandable that the method can also be applied to the terminal. It is applied to include terminals and servers and systems and is realized through the interaction of terminals and servers. The server can be an independent physical server, or a server cluster or distributed system composed of multiple physical servers, or it can provide cloud services, cloud databases, cloud computing, cloud functions, cloud storage, network servers, cloud communications, and intermediate Cloud servers for basic cloud computing services such as software services, domain name services, security services CDN, and big data and artificial intelligence platforms. The terminal can be a smart phone, a tablet computer, a notebook computer, a desktop computer, a smart speaker, a smart watch, etc., but it is not limited to this. The method mentioned in this article includes the following steps:

Semantic-label multigranularity attention model construction: the output of the stacked expanded convolutional coding module and the label graph attention module are connected to the multigranularity attention mechanism network, and the weighted label output by the multigranularity attention mechanism network is used as a full connection. Regarding the input of the layer, the output value obtained by the fully connected layer for mapping the predicted label are input into a Sigmoid layer, and the predicted probability of each label is obtained.

Model training: use the multilabel data set to train the constructed semantic-label multigranularity attention model, adjust the parameters until the semantic-label multigranularity attention model converges, and obtain the trained semantic-label multigranularity attention model; multilabel data set classification: taking the multilabel data set to be classified as input, the semantic-label multigranularity attention model after training outputs the classification result.

In the choice of coding architecture, this paper does not use the traditional CNNRNN or self-attention mechanism but builds the multigranular semantic feature representation of the text sequence hierarchically through the stacked expanded convolution structure. Aiming at the complex correlation between tags, this paper also does not use sequence-to-sequence architecture to generate tag sequences to model but applies a tag graph attention network. It can directly model the label relevance and obtain the updated label representation. In order to efficiently use the semantic information of multiple levels of word phrases and sentences extracted by the encoder, the present invention also designs a multigranularity attention. It uses these types of hierarchical information to weight the label representations, respectively, highlighting the label representations whose semantic features are closely related to the text sequence. Finally, the weighted label representation is sent to a fully connected layer shared with the weight of the label embedding matrix for linear mapping, and a Sigmoid function is used to realize the output of each label probability.

The specific steps of the method proposed in this article are as follows:

The model built in this article consists of four parts: a stacked dilated convolutional coding module, a label graph attention module that models label correlation, a multigranularity attention mechanism, and the weights of the input label embedding matrix with a Sigmoid function, shared fully connected layer.

### 2.1. Stacked Dilated Convolution Module

In this paper, the coding architecture is constructed by continuously stacking the expanded convolution structure, which is used to extract the multigranularity semantic feature representation in the input sequence. For a given word embedding matrix representation,

(1) $$\begin{array}{c} X=\left[x_{1},x_{2},\ldots ,x\right],\\ X=\left[x_{1},x_{2},\ldots ,x_{s}\right],\;X\in R^{S\times d}. \end{array}$$

Unlike standard convolution, which operates on a continuous subsequence of the input sequence at each step, expanded convolution has a wider receptive field by adding 8 holes between words within the subsequence, of which 6 is called the expansion rate. Then, the expansion convolution operation for the center word *x* and the convolution kernel *W* with width *k* can be expressed as

(2) $$\begin{array}{c} c_{i}=\sigma \left(W\overset{k}{\underset{j=0}{⊕}}x_{i\pm j\delta }+b\right) \end{array}$$

where ⊕ is the vector splicing and *b* is the bias term and is the nonlinear activation function. Then, the output of the dilated convolution after the execution of the word vector matrix can be expressed as

(3) $$\begin{array}{c} C=\left[c_{1},c_{2},\ldots ,c_{s}\right], \end{array}$$

where

(4) $$\begin{array}{c} C\in R^{S\times f}. \end{array}$$

In order to maintain the consistency of input and output, the input sequence is zero-filled before the convolution operation, which effectively preserves the semantic information. As shown in Figure 2, the multigranularity semantic information of the input sequence is extracted by stacking expansion convolution. For the first layer, set 8 = 1 (equivalent to standard convolution), so that all words in the input sequence will not be missed. Then, the subsequent stacking of the dilated convolution structure uses a larger dilation rate. The range of the receptive field is expanded in a linear manner, but only a small number of layers and appropriate parameters can cover the entire text sequence.

After each convolutional layer, layer standardization is applied to ensure that the model does not disappear or explode during the training phase. Multilevel expansion rate is designed according to the performance in actual verification. The output of each pair of overlays is a representation of the semantic features of the text at a specific level of granularity. Assuming that the number of stacked layers is *L*, the output of the first stacked layer is

(5) $$\begin{array}{c} C^{l}=\left[c_{1}^{l},c_{2}^{l},\ldots ,c_{s}^{l}\right]. \end{array}$$

where *C* is the number of convolution filters in each layer. The multigranularity semantic features of all stacked layers are expressed as

(6) $$\begin{array}{c} \left[C_{1},C_{2},\ldots ,C_{L}\right]. \end{array}$$

In this way, SDC gradually obtains word-level semantic and local semantic features from the word and phrase level with a small expansion rate and captures the global long-term dependence from the sentence level with a large expansion rate. This coding method not only is superior to traditional sequence models (RNN or LSTM) in parallelism, but also can significantly reduce the amount of parameters and memory loss compared to models based entirely on self-attention mechanisms.

### 2.2. Label Map Attention Module

This paper uses graph attention networks to model the complex dependencies between tags. A label image is composed of label nodes and adjacency matrix. For a data set with a label space size of *L*, the adjacency matrix is constructed on the basis of the entire data set, which can be expressed as AER but is different from using statistical knowledge (frequency or word frequency-inverse document frequency) to loosen fixed weights The parameter label map advocates modeling the correlation between the labels as a weighted map and updates the attention weight and adjacency matrix through the GAT network selective learning method.

The label graph attention network (Label-GAT) takes the label vector obtained through the label embedding matrix WR as input and uses the attention mechanism to participate in the calculation of the weights of neighbor nodes. The calculation process is as follows:

(7) $$\begin{array}{c} h_{t}^{g}=\rho \left(\sum_{r\in N_{t}}\alpha \left(h_{t}^{g-1},h_{r}^{g-1}\right)W^{g-1}h_{r}^{g-1}\right), \end{array}$$

where *α* is the attention function, which adaptively controls the contribution of the neighbor node *r* to the current node *t*. In order to learn the attention weights of different subspaces, a multihead attention mechanism is used in the Label-GAT network.

(8) htg=‖ρm=1M∑r∈Ntαmhtg−1,hrg−1Wmg−1hrg−1.

At the same time, in order to capture the connection between nodes at a greater distance, the Label-GAT network is stacked in multiple layers. The final label representation output through Label-GAT modeling can be expressed as follows:

(9) $$\begin{array}{c} H=\left[h_{1}^{g},h_{2}^{g},\ldots ,h_{L}^{g}\right]. \end{array}$$

### 2.3. Multigranularity Attention Module

It uses the semantic feature representation C at each granularity to weight the label representation *H* output by Label-GAT, thereby highlighting the labels that are closely related to the text sequence.

Inspired by the multihead self-attention mechanism, the semantic feature representation under each granularity is regarded as a different subspace, and the number of subspaces (head number) is the same as that of granularity. By calculating the weights of the label representations in multiple subspaces, the weighted results of all granularities are finally spliced, and the weighted label representations are output.

Assume that *d* represents a Query key-value pair (Key-Value) at the i-th granularity. Then, the output of multigranularity attention at this granularity is

(10) $$\begin{array}{c} H_{\text{attn}}^{l}=\text{softmax}\left(\frac{\left(HW_{q}^{l}\right){\left(C^{l}W_{k}^{l}\right)}^{T}}{\sqrt{d_{k}^{l}}}\right)\left(C^{l}W_{v}^{l}\right). \end{array}$$

Among them, *W* is the weight parameter under the first degree. By aggregating the output at all granularities, the final weighted label is expressed as

(11) $$\begin{array}{c} H_{\text{attn}}=\left[H_{\text{attn}}^{1},H_{\text{attn}}^{2},\ldots ,H_{\text{attn}}^{n}\right]W. \end{array}$$

Among them, *W* is the weight parameter.

### 2.4. Tag Embedded in the Shared Fully Connected Layer

In order to ensure that the embedding representation of each tag corresponds to the feature tag, a fully connected layer that shares the weight of the tag embedding matrix is designed. Specifically, after the model uses W to generate the corresponding label vector, it is again used to map the output value of the predicted label. Subsequently, the output value is fed to a Sigmoid layer to generate the predicted probability of each label:

(12) $$\begin{array}{c} \hat{Y}=\text{sigmoid}\left(W_{y^{\prime }}H_{\text{attn}}\right). \end{array}$$

## 3. Empirical Analysis

In order to simulate the classification of massive digital archive data, 5 types of text data with a large amount are selected for classification experiment; the categories are C19-Computer, C32-Agriculture, C34-Economy, C38-Politics, C39-Sports, and a total of 6 253 texts of data.

In the experiment process, the preprocessing of word segmentation and stop word removal was first performed on the archive data set, and then the five classification category tags were added to the end of the corresponding archive text as the tags of the training data. Put the file training into FastText for deep learning training.

The specific parameters of FastText used in this article are as follows: set the learning rate to 0.1. Considering the efficiency of text classification, the dimension of the word vector is set to 50, which not only ensures the accurate expression of semantics in the text, but also does not excessively reduce the operating efficiency of the algorithm. On the premise that the data set is sufficient, the FastText algorithm only needs 3 full data sets of training to converge, and it has high training efficiency. Regarding semantic level features ngarm = 2, the classifier uses hierarchical Softmax. The important parameter of the FastText model is the context window (ws). The selection of this parameter means the amount of information that can be obtained from the text context sentence. As the size of the context window increases, the F1 value of text classification will also increase, but training time will increase. For the current data set, when the context window value (ws) is 4, the F1 value of each category of the text will stabilize, reaching about 0.96. In this experiment, FastText model, Naive_Bayes (naive Bayes) model, and SVM model are used for classification training respectively, and the above-mentioned test set is used to verify the classification results. The classification results of the three types of models are shown in Figure 3. According to the evaluation criteria of machine learning classification, the precision rate, recall rate, and *F*1 value of each of the 5 types of text data are, respectively, obtained, and the macro average, micro average, and weighted average precision rate, recall rate, and recall rate of the comprehensive text test set are calculated. F1 value displays the number of test files of each type at the same time.

The FastText model performed stably in the testing of the test set. In the multiclassification experiment with a total of 6 253 files, the classification accuracy, recall, and *F*1 value of each category were maintained above 0.94, as shown in Figure 3(a). The performance of the Naive_Bayes model in the test set fluctuates slightly. In the multicategory with a total of 6 253 files, the accuracy, recall and F1 value of each category are maintained above 0.92, as shown in the Figure 3(b). The SVM model performed poorly on the test set. In the multicategory with a total of 6 253 files, the accuracy, recall, and *F*1 value of each category are quite different, and the lowest can only reach 0.52, as shown in Figure 3(c). The predicted also can be found in Figure 4.

Since most of the archive text data is clear, and there is a need for classification and archiving, it is suitable for automatic classification using deep learning. In this experiment, the classification accuracy of the FastText-based text classification model in the three categories of C19-Computer, C32-Agriculture, and C34-Economy is higher than that of the Naive_Bayes model, and the classification of the two categories of C38-Politics and C39-Sports The accuracy is the same as that of the Naive_Bayes model. The reason for this is because the content of the data set used in the experiment is clear, and the original text features are enough to make the Naive_Bayes model make accurate classification judgments. Even so, the FastText-based classification model in this article can also win in some data categories, which proves the effectiveness of the FastText-based classification model in text classification. The advantage of this classification accuracy will increase with the complexity of the archive data set, which is more prominent.

At the same time, the accuracy of the FastText-based text classification model in all categories is much higher than that of the SVM-based text classification model. From the perspective of the mathematical model, the hyperplane formed by the SVM is not suitable for the text features of the file subject. Although the model is simple, the efficiency of the model is acceptable, but there is still a gap in accuracy compared with the model based on FastText.

It can be seen from Figure 5 that, in the five categories of classification verification experiments, the FastText-based text classification model has reached the classification F1 values on C19-Computer, C32-Agriculture, C34-Economy, C38-Politics, and C39-Sports as 1.00, 0.95, 0.94, 0.95, and 0.97. It can be seen from the above figure that the weighted *F*1 value of the naive Bayes classifier is 0.95, and the F1 value of the SVM classifier is 0.73. The text classification model based on FastText is in terms of weighted *F*1 value, weighted average precision rate, and weighted average recall rate. Among the three overall category evaluation indicators, it is far superior to the text classifier based on the SVM model, which is about 1% improvement over the text classification model based on Naive Bayes, and the overall evaluation F1 value has reached 0.96, basically replacing the manual level of classification.

The label space is fixed to *n*. Using the transfer method can effectively reduce the label space (from 2*n* to *n*), reduce the computational complexity, and compress the training time. The experimental strategy is to use single-label data for training and verification and use multilabel data or all data for testing. Therefore, Reuters-21578 was reprocessed, and two sets of experiments were designed. Reuters-Multilabel and Reuters-Full remove all multilabel data in the training set and validation set, leaving only 5912 single-label data. Reuters-Multilabel retains only 437 multilabel data in the test set; Reuters-Full contains all 3019 data.

A comprehensive comparison is made between the proposed model SLMA, capsule network, and SGM. Use MicroF1 score and MacroF1 score as evaluation indicators instead of Hamming loss. In addition, we have introduced precision (Precision) and recall (Recal1) for a more comprehensive comparison. The results show that, on the test sets of the Reuters-Multilabel and Reuters-Full data sets, our method has significant advantages over Capsule and SGM in all four evaluation indicators. Especially on the Reuters-Multilabel dataset, which only contains multilabel data, a great improvement has been made in the testing process. Different from the capsule network, SLMA and SGM focus on predicting tags through the content of different positions in the text, instead of using document-level prediction. SLMA provides a multigranular semantic feature representation that can take into account local semantics and long-term dependence through a stacked expanded convolution structure. It provides richer and finer-grained text information for label prediction, so it is better than SGM in performance. In addition, the good results when using Reuters-Full data for testing also show that SLMA has a strong advantage over competitors in single-label data. Experiments on the robustness of the model when faced with high and low-frequency data: in the experimental results of the above data set, it is observed that the performance of SLMA on low-frequency tags is not as good as high frequency. The *y* versus *x* is shown in Figure 6.

Consistent with the prediction, the ratio of the overall sample size to the internal label data caused the performance difference of the model on different label frequencies. In order to observe the overall performance of SLMA more intuitively, two sets of experiments are set up, using MicroF1 and MacroF1 to measure the performance of high-frequency and low-frequency tags, respectively. In addition, for the convenience of comparison, SGM is also used to evaluate RCV1-V2. For the model performance of high-frequency tags, the 10, 20, 30, 40, 50, and 60 tags with the lowest frequency are eliminated. For low-frequency tags, remove the 10, 20, 30, 40, 50, and 60 tags with the highest frequency.

Figure 7 is the results of SLMA and SG on high-frequency and low-frequency tag data. But in the case of tag frequency changes, the SLMA model still maintains a better performance than the strong baseline SGM, and the gap is gradually widening. In contrast, despite the reduction of high-frequency tags, the performance of the two models has different degrees of decline, but our proposed SLMA is more robust than SGM in classifying low-frequency tags. Compared with Seg2Sea-based SGM, SLMA gets rid of the dependence on the order of tag frequency (descending or ascending) and pays more attention to the connection between the multigranular semantic representation of the text and the tags from the perspective of local semantics and long-term dependence. Not only does it perform well in high-frequency tags, but it also more robustly classifies low-frequency tags.

In summary, for multilabel text classification tasks, a semantic-label fine-grained attention model with strong interpretability is proposed. This model constructs a multigranular semantic feature representation of the text sequence in terms of local relevance and long-term dependence through the stacked expanded convolution structure. We conducted a series of experiments on three benchmark data sets, and the results show that the proposed model has very advanced performance in various evaluation indicators. Additional analysis experiments show that our model not only has good migration ability, but also shows strong robustness in the face of high and low-frequency data.

## 4. Conclusion

This paper proposes an intelligent classification method for archive data based on multigranular semantics. The first is to construct a semantic-label multigranular attention model; that is, the output of the stacked expanded convolutional coding module and the label graph attention module are connected to the multigranular attention mechanism network. The weighted label output by the multigranular attention mechanism network is used as the input of the fully connected layer, and the output value of the fully connected layer used to map the predicted label is input into a Sigmoid layer to obtain the predicted probability of each label; then, the model is trained. Use the multilabel data set to train the constructed semantic-label multigranularity attention model, adjust the parameters until the semantic-label multigranularity attention model converges, and obtain the trained semantic-label multigranularity attention model. Taking the multilabel data set to be classified as input, the semantic-label multigranularity attention model after training outputs the classification result.

The research basis of this paper is predefined rules. However, the research on predefined rules is not perfect, and a unified definition of rules has not been formed. We can make an in-depth analysis in this aspect in the future.

## Figures and Tables

**Figure 1:** Multilabel classification method.

**Figure 2:** The multigranularity semantic information.

**Figure 3:** Results of classification. (a) FastText, (b) Naive_Bayes, and (c) SVM.

**Figure 4:** Predicted value.

**Figure 5:** Five categories of classification verification experiments.

**Figure 6:** *y* versus *x*.

**Figure 7:** The results of SLMA and SG. (a) High frequency. (b) Low frequency.

## Data Availability

The dataset can be accessed upon request.
